This article has been retracted.

# Production of Gymnemic Acid Depends on Medium, Explants, PGRs, Color Lights, Temperature, Photoperiod, and Sucrose Sources in Batch Culture of *Gymnema sylvestre*

**DOI:** 10.1100/2012/897867

**Published:** 2012-05-02

**Authors:** A. Bakrudeen Ali Ahmed, A. S. Rao, M. V. Rao, Rosna Mat Taha

**Affiliations:** ^1^Institute of Biological Sciences, Faculty of Science, University of Malaya, 50603 Kuala Lumpur, Malaysia; ^2^Department of Plant Science, Bharathidasan University, Tamil Nadu, Tiruchirappalli 620 024, India; ^3^Department of Biotechnology, Bharathidasan University, Tamil Nadu, Tiruchirappalli 620 024, India

## Abstract

*Gymnema sylvestre* (R.Br.) is an important diabetic medicinal plant which yields pharmaceutically active compounds called gymnemic acid (GA). The present study describes callus induction and the subsequent batch culture optimization and GA quantification determined by linearity, precision, accuracy, and recovery. Best callus induction of GA was noticed in MS medium combined with 2,4-D (1.5 mg/L) and KN (0.5 mg/L). Evaluation and isolation of GA from the calluses derived from different plant parts, namely, leaf, stem and petioles have been done in the present case for the first time. Factors such as light, temperature, sucrose, and photoperiod were studied to observe their effect on GA production. Temperature conditions completely inhibited GA production. Out of the different sucrose concentrations tested, the highest yield (35.4 mg/g d.w) was found at 5% sucrose followed by 12 h photoperiod (26.86 mg/g d.w). Maximum GA production (58.28 mg/g d.w) was observed in blue light. The results showed that physical and chemical factors greatly influence the production of GA in callus cultures of *G. sylvestre*. The factors optimized for *in vitro* production of GA during the present study can successfully be employed for their large-scale production in bioreactors.

## 1. Introduction

*In vitro* techniques are very useful in ensuring sustainable, optimized sources of plant-derived natural products. However, *ex situ* cultivation should be preceded by proper evaluation of the plants for their ability to produce the required bioactive constituents before commencing cultivation or introducing the technology to potential growers. The ability of plants to produce certain bioactive substances is largely influenced by the physical and chemical environments in which they grow. Plants also produce certain chemicals to overcome abiotic stresses [1]. Plants use light not only as an energy source for photosynthesis but also as an important environmental signal. Plants can detect almost all facets of light such as direction, duration, quantity, and wavelength by using three classes of photoreceptors: the red/far-red (600–750 nm) absorbing phytochromes, and the blue/UV-A (320–500 nm) absorbing cryptochromes. These photoreceptors perceive, interpret, and transducer light signals, via distinct intracellular signaling pathways, to mediate a broad range of physiological responses to light in addition to cell growth and development [2]. Light can affect morphogenesis and the formation of plant metabolites as a signal and stress factor from phytohormones. In most plant cell cultures, secondary metabolism, including the production of phenolic terpenoid and alkaloid compounds, is stimulated by light [3]. On the other hand, light had an inhibitory effect on the accumulation of secondary metabolites in the case of nicotine and shikonin [4]. The literature shows that the majority of pharmacologically important compounds of plant origin are products of defense and secondary metabolism [1, 5]. This ability of plants to respond to physical and/or chemical stimuli can be used for elicitation of pharmacologically active substances by subjecting an intact plant to stress factor(s) [1]. Growing a plant outside its natural environment under ideal conditions may therefore, result in it being unable to produce the desired bioactive substance, hence the need for prior evaluation.

*Gymnema sylvestre *is an important medicinal climber belonging to the family Asclepiadaceae. This climber is extensively used in almost all the Indian systems of medicine as a remedy for rheumatism, cough, ulcer, and pain in the eyes. It is also useful for inflammations, dyspepsia, constipation, jaundice, and so forth. The roots of this plant have been reported as a remedy for snakebite [6]. The plants occur mainly in the Deccan peninsula of western India, Tropical Africa, Vietnam, Malaysia, SriLanka and is widely available in Japan, Germany, and the USA as a health food [7]. The extract of *G. sylvestre* plays a major role in blood glucose homeostasis through increased serum insulin level through regeneration of the endocrine pancreas [8]. We have reported that leaf and callus extracts of *G. sylvestre* maintained the blood glucose and lipid profiles in alloxan-induced diabetic Wistar rats [9]. Several research studies in the early 2000s described *G. sylvestre* callus culture for the production of GA. Physical stress was established in which MS medium supplemented with PGRs was used for callus growth, and modifying the shaking speed, pH and medium play an important role in the production of GA [10]. Furthermore, Lee et al. (2006) tried the addition of sucrose, inoculum density, and aeration factors suitable for GA production by using bioreactors [11]. Veerashree et al. (2012) reported that yeast extract, pectin, and chitin elicitor enhanced the GA via cell suspension culture [12]. We have recently reported the *G. sylvestre in vivo* and *in vitro* callus extracts regenerated the damaged pancreatic *β* cells in alloxan-induced diabetic Wistar rats [13]. The present study highlights the evaluation of GA content in: (i) callus derived from different plant parts of *G. sylvestre*, namely leaves, stem and petioles; (ii) *in vitro* elicitation of GA employing physical-chemical factors of light, temperature, photoperiod, and sucrose concentration; (iii) isolation and characterization of GA from callus, namely, HPTLC and HPLC.

## 2. Materials and Methods

### 2.1. Chemicals

Standard GA was gifted by Professor Kazuko Yoshikawa, Department of Pharmaceutical Science, Kyoto Pharmaceutical University, Japan. Medium salt bases and adenine sulphate were purchased from Sigma Chemical Co., USA. Other medium components and phytohormones were of tissue culture grade or equivalent. All solvents used for chromatographic purposes were HPLC grade. Other solvents were reagent grade or equivalent.

### 2.2. Plant Material and Sterilization

*G. sylvestre* was collected from the Pachamalai hills (attitude: 1000–1200 m), Tamil Nadu, India, and maintained in the Department of Plant Science garden of the Bharathidasan University, Tiruchirappalli, Tamil Nadu, India. Healthy, young leaf, stems (shoot internodal segment without buds), and petiole explants (Figure 1(a)) were washed thoroughly in running tap water 3–5 times, including 2% (v/v) Teepol (Reckitt Benckiser, India) for 10 min, then washed with 70% ethanol for 30 sec followed by another wash with 0.1% HgCl_2_ for 2 min. Prior to inoculation, the explants were washed three times with distilled water.

### 2.3. Callus Induction and Culture Conditions

Leaf, stem, and petiole explants of *G. sylvestre* were grown in MS medium [14], SH medium [15], B5 medium [16], and WPM [17] (woody plant medium) supplemented with 0.5–5.0 mg/L of IAA (indole-3-acetic acid), IBA (indole-3-butyric acid), NAA (1-naphthaleneacetic acid), 2,4-D (2,4-dichlorophenoxyacetic acid); 0.2–2.0 mg/L of BA (6-benzylaminopurine) and KN (6-Furfurylaminopurine) were used for callus induction. The callus culture was maintained at 25 ± 2°C, 16/8 h (light/dark) of photoperiod with 25 *μ*mol m^−2^ s^−1^ of light intensity. The pH of the medium was adjusted to 5.7–5.8 and gelled with 0.8% agar (w/v) (Bacteriological grade, Hi-media, India). Sucrose 30 g/L (Hi-media, India) served as the carbon source. The culture medium was sterilized by autoclaving at 1.06 kg cm^−1^ and 121°C for 20 min. The role of media on the nature and biomass of callus was studied in leaf, stem, and petiole explants of *G. sylvestre*.

### 2.4. Measurement of Callus Growth

For all callus growth measurement experiments, 40 mg fresh weight of leaf (*in vivo*) was inoculated on to 20 mL of the fresh agar MS solid medium in the culture tube (25 × 150 mm), and the biomass gain was monitored at 10 day intervals over a 0–55-days cultured cycle. By treating with various combinations of auxins and cytokinins, fresh and dry weights of the calli were determined at 0–15, 15–25, 25–35, 35–45, and 45–55 days. At regular intervals for all treatments, each callus was harvested by careful separation from the media using metal spatulas, and fresh and dry weight was promptly recorded. A minimum of 3 replicates were run for all the treatments, and the experiments were repeated thrice.

### 2.5. Physical-Chemical Stress Condition

For improvement of GA, *G. sylvestre* callus cells, 15–25-day-old cells, were placed in the different physical stress of lights (blue, red, green, and white fluorescent tube, Phillips, India); temperature (20°C, 25 ± 2°C, 30°C, and 35°C); photoperiod (4 h/20 h, 8 h/16 h, 12 h/12 h, and 20 h/4 h light/dark) and chemical stress of sucrose (2%, 4%, 5%, and 6%), respectively. OPGRs [MS + 2,4-D (1.5 mg/L) + KN (0.5 mg/L)], 25 ± 2°C, 16 h/8 h (light/dark), 3% sucrose kept under white fluorescent tube used as control. All treatment callus biomass was determined using growth curve analysis, in all the physical-chemical treatments. After treatment, callus cells were harvested at time intervals, washed twice with 100 mL water on a porous glass funnel with filter paper (Whatman No-1), then frozen in liquid nitrogen, and stored in the deep freezer for further investigation and analysis.

### 2.6. GA Extraction and Phytochemical Analyses

The extraction, sample preparation, and chromatographic analyses (HPTLC and HPLC) were performed. Briefly, *in vivo* leaf and *in vitro* callus (500 mg d.w) were extracted with methanol 5 times as described by Rehman et al. [18]. The collected methanol extract was centrifuged at 5000 × g for 10 min at room temperature, and then the methanol supernatant was carefully pipetted out into fresh eppendorf tubes without disturbing the inter-phase residues. Green-color methanol supernatant (4 mL) was evaporated and dried. The residue (ca. 6 mg) was dissolved in MeOH (5.0 mL) and 20 *μ*L injected on HPTLC and HPLC with standard GA. HPTLC system (Camag, Switzerland) assisted with sample applicator Linomat IV for quantification of GA. 10 samples were applied on each plate at a start line 8 mm from the bottom, including nine lanes of *in vitro* callus and *in vivo* leaves with standard GA (20 *μ*L). The mobile phase of isopropyl alcohol : chloroform : methanol : acetic acid (5 : 3: 1 : 0.5; v/v/v/v) was allowed to run up to 80 mm for separation of GA at a wavelength of 200 nm by the use of TLC scanner III, integration and quantification was performed using CAT 4.0 software.

 Methanol extracts of *in vivo* leaf and *in vitro* callus were further analyzed via HPLC (Shimadzu, Kyoto, Japan). This system consisted of a two 510 Pumps, a 7725 Rheodyne auto injector, a DUG-12 A degasser, SCL-10Avp system controller, C_18_ (ODS) reverse-phase column (150 mm × 4.6 mm i.d., 5 *μ*M particle size), and a Spectromonitor 486 variable wavelength UV/VIS detector. The analog detector output was acquired and digitized by an Advanced Computer Interface and then processed by AI-450 Chromatography Automation Software (Dionex Corp., Sunnyvale, CA, USA). The flow rate used was 1.0 mL/min, and GA was detected by UV absorption at 230 nm with a mobile phase of 0.1% acetic acid, 35% water, and 65% methanol (HPLC grade). Each injection volume was 20 *μ*L. For quantification of GA, the respective retention time (*R*_*T*_) and peak area were calculated.

### 2.7. Method Validation

#### 2.7.1. Linearity

In this study, each calibration curve was analysed three to times with three to four different concentrations using the same HPLC condition as described above. The calibration graphs were plotted based on linear regression analysis on the integrated peak areas (*y*) versus concentrations (*x*). The regression equation was calculated in the form of *y* = *ax* + *b*, where *y* and *x* were the values of peak area and sample amount, respectively. The standard solution was diluted with methanol to provide appropriate concentrations. The limit of detection (LOD) was defined as the lowest concentration level resulting in a peak area of three times the baseline. The limit of quantification (LOQ) was defined as the lowest concentration level resulting in a peak area of ten times the baseline.

#### 2.7.2. Precision

The precision test was evaluated by the intra-day and inter-day variability. Three different concentration solutions (low, medium and high) of the standards were prepared in methanol. Three replicates of the samples at each concentration were evaluated on the same day for intra-day precision, whilst repeated analysis at each concentration of the samples three times per day over three consecutive days for inter-day precision. The quantity of each analyte was obtained from corresponding calibration curve. The relative standard deviation (R.S.D) was taken as a measure of precision.

#### 2.7.3. Recovery

In order to check the accuracy of the developed method, the recovery experiments were carried out as follows: three different quantities (low, medium and high) of the authentic standards were spiked into the samples in form of solution. The quantity of each analyte was subsequently obtained from the corresponding calibration curve.

### 2.8. Statistical Analysis

All the experiments were repeated thrice and 30 replicates were used. The effect of different treatments was quantified as mean ± SE and the data were subjected to statistical analysis using Duncan's multiple range test (DMRT) at 5% level significance [19].

## 3. Results and Discussion

### 3.1. Influence of PGRS, Medium and Explants on Callus Induction

In all the media tested, the callus initiation did not occur without PGRs (control) in leaf explants of *G. sylvestre*. The suitable callus induction was obtained in 2,4-D and NAA on MS, B5, SH and WPM medium which induced GCC (green compact callus), GFC (green friable callus), WFC (white friable callus), WWC (white watery callus) and BFC (brown friable callus) in leaf, petiole and stem explants. For successful callus induction, factors such as type of explants, PGRs, culture media and cultural conditions are very important [20]. MS medium callus induction, proliferation and biomass (fresh and dry weight) was better than B5, SH and WPM medium (Figures 1(b)–1(e); 2(a)–2(h)). The leaf explants produced GCC with higher induction frequency (94.5%) than petiole (79.1%) and shoot tip explants (72%) cultured on MS medium (Figures 1(f)–1(h); 3(a)–3(d)). Among the various concentrations of auxins tried in callus induction, 2,4-D (1.5 mg/L; 93.5%) and NAA (1.0 mg/L; 86.8%) significantly induced GC natured callus with a maximum biomass at 35–45 days in terms of fresh and dry weight (Figures 2(a)–2(d)). In our study, callus biomass progressively increased with an increase in the 1.5 mg/L of 2,4-D (GCC; DW-121 mg/L; Figure 1(i)) and 1.0 mg/L of NAA (GCC; DW-115 mg/L; Figure 1(j)) concentration (>0.5–1.5 mg/L) especially when the culture contains NAA concentration of 2.5–5.0 mg/L, WFC and WWC were induced significantly. In addition, it was observed that 1.5 mg/L of IBA (DW-87 mg/L; Figure 1(k)) and 2.0 mg/L of IAA (DW-63 mg/L; Figure 1(l)) and drastically reduced the callus biomass resulting in WFC natured calli all the media. These results are well authenticated with previous reports of Rani et al. (2010), who demonstrated that NAA and 2,4-D were suitable for the callus induction of *G. sylvestre* [21]. 

Successful biomass was obtained by the use of 2,4-D (1.5 mg/L) with BA (0.5 mg/L) (DW-113 mg/L; Figure 1(m)) and 2,4-D (1.5 mg/L) and KN (0.5 mg/L) (DW-144 mg/L; Figure 1(n)), which increased GC nature at 35–45 days. However, 2,4-D + BA and 2,4-D + KN (<3.0–5.0 mg/L) combinations drastically reduced the callus biomass and showed the GFC, BFC, and WFC (data not shown). Auxins and cytokinins regulate plant cell division, which influenced the different phases of the growth cycle and regulates the signalling pathway [22]. In addition, various combinations of NAA with BA, and KN were tried for callus biomass, which resulted in less biomass and GC nature than 2,4-D with BA, and KN (data not shown). During the callus biomass, the batch callus culture was continuously examined by taking a subculture at weekly intervals to prevent cell death and browning of media. 

### 3.2. Measurement of Callus Growth Curve

*G. sylvestre* callus growth curve was sigmoid, and four growth phases can be distinguished in the MS medium supplemented with OPGRs [2,4-D (1.5 mg/L) + KN (0.5 mg/L)] at different days (0–15, 15–25, 25–35, 35–45, and 45–55 days). In the lag phase (0–15 days; DW-49 mg/L), *in vitro* callus was slowed at the initial stage; the callus biomass was drastically reduced over the other phase, and the GA content was absent (data not shown). In the lag phase (15–25 days; DW-92 mg/L), callus initiation and proliferation were observed by profound cell division [23]. At 25–35 days (exponential phase), biomass (DW-105 mg/L) of the GC was significantly increased. The MS medium supplemented with OPGRs induced the high level of callus biomass in the stationary phase (35–45 days; DW-144 mg/L; Figure 1(o)) of the callus growth curve suggests the cellular membrane stabilization. It has been previously reported that the stationary phase callus evidently demonstrated an increase in the accumulation of gagaminine in the callus (GC) of *Cynanchum wilfordii* [24]. At the decline phase (45–55 days; DW-119 mg/L), the callus biomass was drastically reduced as compared to other phases.

### 3.3. Influence of Color Light on Callus Induction

Light is an important physical factor, which influences growth, development, and the formation of primary and secondary metabolites [25]. In the present study, color light was also one of the most important factors in inducing and maintaining GC nature of the cells on *G. sylvestre* callus (Figure 4(d)). The analysis of *G. sylvestre* callus growth in batch culture under blue light conditions showed that GC callus yielded higher biomass (DW-172 mg/L) at the stationary phase of 35–45 days of culture (Figure 4(a)). In general, the optimal flux of blue light for leaf explants is about 10–15% of the total photosynthetically active radiation. Moreover, the higher flux of blue light is essential for normal carbohydrate metabolism, photosynthetic assimilating, and transport from leaves. Cryptochrome wave length (450 nm), was closed to the blue light, and in this condition more Pr transformed into Pfr for phenylethanoid glycoside production [26]. Figure 4(b) callus growth on red light was, however, extremely slow, and growth curve values of only 31 mg/L, 59 mg/L, 85 mg/L, 122 mg/L and 102 mg/L of dry weight could be registered after 15, 25, 35, 45, and 55 days of the growth. In comparison, MS medium + OPGRs with green light supported maximum GA accumulation in callus harvested on 35–45 days of incubation, respectively, (DW 116 mg/L; Figure 4(c)).

### 3.4. Influence of Temperature on Callus Induction

Temperature has many effects on the mechanisms of metabolic regulation, permeability, nutritional needs, and the rate of intracellular reactions in plant cell cultures [27]. 30°C increased the callus biomass and decreased the GA content (2.9 mg/g d.w) than the control (25 ± 2°C) in 35–45 days of stationary phase. Thus, changing the culture temperature may change the physiology and metabolism of cultured cells and subsequently affect callus growth and secondary metabolite production. The callus culture exposed to the lower temperature (20 ± 2°C) showed decrease in callus biomass (DW-45 mg/L) and GA content (0.03 mg/g d.w) (Figure 4(e)). MS medium supplemented with OPGRs kept under 30°C induced GFC (Figure 4(f)) and biomass (DW-150 mg/L) in *G. sylvestre*. However, each plant species may favour a different temperature. For strawberry callus culture, maximum anthocyanin content was obtained at 15°C and it was about 13 fold higher than that obtained at 35°C [27]. The cultures incubated at 35 ± 2°C had lower callus biomass (DW-125 mg/L) and GA (1.4 mg/g d.w) (Figure 4(g)), respectively. For Asclepiadaceae species, callus biomass increased at 31°C, more than at 25°C, hence gagaminine content was higher at 25°C in* Cynanchum wilfordii* [24].

### 3.5. Influence of Sucrose on Callus Induction

GA productivity at the growth stage (35–45 day) was also assessed at seven concentrations of sucrose (1–6% w/v) under continuous illumination. Data showed that the OPGRs biomass increase in selected callus line was highest at 5% level of sucrose after 35–45 day of culture (DW-164 mg/L; GA content 33.3 mg/g d.w; Figure 4(h)). Kintzios et al. (2003) reported that MS medium supplemented with auxins and cytokinins in combination to treatment of 5% sucrose induced the rosmarinic acid in* Ocimum basilicum* [28]. Cultures grown on MS medium with 1.0% sucrose indicated a further drastic fall in biomass in all the growth phases (data not shown). GA production, on the other hand, was found to be positively correlated with increasing sucrose concentration in the medium up to 3.0% after 45 days (control) and GA content (12.77 mg/g d.w). We have found that GA content depends on the callus biomass in sucrose treatment. The lowest GA content was recorded in tissue cultured on 2.0% (biomass DW-89 mg/L; GA-5.4 mg/g d.w; Figure 4(i)), 4.0% (biomass DW-152 mg/L; GA-17.6 mg/g d.w; Figure 4(j)), 6.0% (biomass DW-108 mg/L; GA-24.1 mg/g d.w; Figure 4(k)) at 35–45 days of stationary phase, respectively. When data on biomass gain and GA contents were extrapolated in terms of net GA yield, it was found that cultures grown in presence of 1.0–6.0% sucrose supplementation had almost different levels of GA until day 55 of the culture cycle. However, if the culture cycle was extended to 65 days, then cultures on medium with 7-8% sucrose were lesser yielders of the GA and callus biomass (data not shown).

### 3.6. Influence of Photoperiod on Callus Induction

Influence of photoperiod on callus growth and GA accumulation was also studied under seven sets of lights and dark regimes: (a) 4 h light/20-h dark, (b) 8 h light/16 h dark, (c) 12 h light/12 h dark, (d) 16 h light/8 h dark (control), (e) 20 h light/4 h dark, (f) 24 h light, (g) 24 h dark. A time course study at 10 day intervals under the 12 h light/12 h dark photoperiod conditions indicated that selected OPGRs callus attained maximum biomass gain (DW-159 mg/L; GA-26.27 mg/g d.w; Figure 4(l)) on the 35–45th day of culture under continuous light conditions. Zhang et al. (1995) succeeded in 12 h light/12 h dark photoperiod with MS medium increased the triterpenoids of harringtonine, homoharringtonine, and isoharringtonine via batch culture in *Cephalotaxus fortunei* [29]. Rapid biomass gain in these cultures became evident between 15th and 45th day, followed by slight decline around the 55th day of the culture cycle. In the present study, less callus biomass was produced in 4-h light/20-h dark (DW-59 mg/L; Figure 4(m)), 24-h light (DW-35 mg/L; Figure 4(n)), and 24-h dark (DW-45 mg/L; Figure 4(o)), when compared to 8-h light/16-h dark (DW-132 mg/L; Figure 4(p)). Incubation in complete darkness resulted in poor callus growth during the initial 15–55 days of the culture cycle. 

### 3.7. Screening and Quantification of Gymnemic Acid

For TLC separation, the intact leaf and callus extracts reaction mixtures were applied to the plates after concentrating. IAA and IBA induced callus extracts that did not show the brown band in TLC and HPTLC analysis, when sprayed with the vanillin sulphuric acid reagent. PGRs (combination of auxins and cytokinins) methanol extracts showed brown bands and the Rf value close to the standard GA. When the auxins and cytokinins concentrations were increased; the plant cells induced the brown friable, white friable, and white compact callus extracts Rf values were slightly higher than the green compact callus (data not shown).

The developed TLC plates were scanned for several times with the same parameters. The concentrates (x 10) callus extract samples were analyzed in one run, this method proves to be very sensitive, relatively fast, inexpensive, and suitable for therapeutic drug monitoring and pharmacokinetic studies [30]. The chromatography developing time was shorter in HPTLC (6 min) than in TLC (40 min) of the mobile phase of Isopropyl alcohol: chloroform: methanol: acetic acid (5 : 3 : 1 : 0.5; v/v/v/v). The gifted GA purity was confirmed in the leaf and callus extracts by recording the absorption spectra at the start, middle, and end of the peak. Standard GA had shown the single peak at different time intervals of the experiment. The intact leaf and callus extracts sample curve was linear; the correlation coefficients had good linearity between concentration and area, it could be helpful to calculate the GA amount in the respectable sample. Green friable callus was induced in MS medium supplemented with NAA (1.0 mg/L) and 2,4-D (1.5 mg/L), and the GA content was drastically reduced with the combination of auxins and cytokinins. When, NAA and 2,4-D are combined with cytokinins, the callus extracts increased the GA content. This controversial MS medium with OPGRs only has produced the maximum biomass and GA compared to the combinations of auxins and cytokinins in 35–45 days of the stationary phase. GA was significantly increased in the MS medium combined with auxins and cytokinins where concentrations derived from leaf explants of *G. sylvestre *were determined in HPTLC [31].

For the HPLC analysis, leaf and callus methanol extracts (20 *μ*L) were uploaded in the HPLC system to quantify GA under retention time (5 min) with help of UV spectrophotometer where peak area data was compared with standard GA. Secondary metabolites were increased in callus culture of *G. sylvestre* [12, 13, 21, 32]. Maximum GA production was observed in MS medium supplemented with OPGRs under blue light-induced 4.4-fold as compared with white fluorescent light and out of which 2.8-fold is found in intact leaves determined by HPLC analysis. We have recently published a paper of pharmacological activities, a phytochemical investigation and *in vitro* studies of *G. sylvestre* [33].

In the HPLC mobile phase [0.1% acetic acid; water/methanol (v/v) (35 : 65, HPLC grade)], purity was analyzed, without sample and with standard GA (Figure 5(a)). Standard GA stability and impurity were characterized through single peak at initial, middle, and end of the HPLC experiment. Imoto et al. (1991) reported that GA content was confirmed through HPLC in methanol leaf extracts of *G. sylvestre* [34].  Figure 5(b) describes the GA content of in intact leaf explants (19.52 mg/g d.w), which was increased compared to Figure 5(c) of *in vitro* callus culture of MS medium supplemented with OPGRS (12.22 mg/g d.w). Many authors had isolated and identified GA earlier in leaf explants of methanol extracts. In 1989, Yoshikawa and coworkers isolated GAs from a hot water extract of *G. sylvestre*, which they named GA I, II, III, IV, V, VI, and VII, respectively, and evaluated using HPLC [35, 36]. For GA enhancement, OPGRs culture was kept under physical-chemical stress conditions determined by growth curve analysis. Blue light with OPGRs induced the maximum GA (53.94 mg/g d.w) (Figure 5(d)) rather than 5% sucrose treatment (33.39 mg/g d.w). However, with other physical stress conditions, the GA was reduced in this order 12 h photoperiod (26.27 mg/g d.w), red light (8.90 mg/g d.w), green light (5.72 mg/g d.w), and 30°C (2.9 mg/g d.w). In case of dark treatment, GA content was absent. We have reported, that *in vitro* callus of *G. sylvestre* significantly increased the pancreatic *β*-cells and maintained the body weight, pancreas weight, liver weight and liver glycogen level in alloxan-induced diabetic Wistar rats [13].

### 3.8. Linearity, Precision, Recovery, and Robustness in HPLC

As per the ICH guidelines, the method validation parameters checked were linearity, accuracy, precision, limit of detection, limit of quantification, and robustness. The linearity of the method was determined at three concentrations (10–30 ug/mL) of GA. 20 ug/mL GA results show that an excellent correlation exists between response factor and concentration of GA within the concentration range indicated above.

The accuracy of the method was determined by recovery experiments. The recovery studies were carried out at three levels of 80, 100, and 120%, and the percentage recovery was calculated. Our studies recovery was within the range of 100 ± 2% which indicates accuracy of the method. The precision of the method was demonstrated by interday and intraday variation studies. In the intraday studies, 3 repeated injections of standard and sample solution were made in a day and the response factor of GA peaks and percentage were calculated. In the interday variation studies, 3 repeated injections of standard and sample solutions were made on 3 consecutive days, and response factor of GA peak and percentage were measured. Intra- and interday accuracy were established from quality control standards by evaluating nominal and mean measured concentrations of quality control standards which were compared and expressed as % difference (diff %). Diff % was calculated using the formula: Diff % = [(mean measured concentration − nominal concentration)/nominal concentration] × 100.

Wave length (200 nm) GA compound was studied showing that a sufficient absorption and an overloading of the column can be avoided. Adding 0.2% acetic acid gave a rather good separation of GA. In order to shorten the analytical time and improve the sensitivity and peak shape of GA a gradient, characterized by an decreased amount of acetic acid (0.1%), was applied before the elution of GA. However, GA is eluted isocratically in order to guarantee robustness.

In conclusion, the present research has provided new information about *in vitro* secondary metabolites, especially the effects of light, temperature, sucrose, and photoperiod. Enhancement of bioactive compounds through different physical and chemical factors has been achieved at all levels. (i) Our study on batch culture of leaf explants of *G. sylvestre* has shown that both the biomass and GA accumulation were influenced by the OPGRs with blue light stress. (ii) Growth curve analysis, GA production and biomass were higher in the stationary phase of all treatments at 35–45 days. Although precise mechanism as to how these factors affect GA remains to be determined, a combination of these factors used for production of valuable compounds via *in vitro* abiotic stresses in the future is a promising strategy. In addition, a simple, reliable, and accurate HPLC assay method of simultaneous determination of GA from *G. sylvestre* was successfully established. The above results will be useful in designing systems for the large-scale cultivation for the production of GA.

## Figures and Tables

**Figure 1:** Effect of culture media, explants, and PGRs on callus induction in *Gymnema sylvestre* after 45 days. (a) Habit; (b) B5 medium (1.2x); (c) SH medium (1.3x); (d) MS medium (1.3x); (e) WPM medium (1.4x); (f) petiole (1.2x); (g) stem (1.3x); (h) leaf explants (1.2x); (i) 2,4-D treatment (2.1x); (j) NAA treatment (1.5x); (k) IBA treatment (1.5x); (l) IAA treatment (2.5x); (m) 2,4-D + BA (1.5x); (n) 2,4-D + KN (1.5x); (o) mass callus culture.

**Figure 2:** Effect of different media (B5, MS, SH, and WPM) supplemented with 2,4-D and NAA on induction of biomass (fresh and dry weight) on leaf explants after 45 days of incubation.

**Figure 3:** Effect of MS medium supplemented with auxins and petiole, leaf, stem explants role on callus induction (%) of *Gymnema sylvestre *after 45th day of incubation.

**Figure 4:** MS medium supplemented with OPGRs, physical and chemical treatments on leaf explants of *Gymnema sylvestre* induced callus after 45 days incubation. (a) Blue light (1.8x); (b) red light (1.8x); (c) green light (1.6x); (d) color light setup; (e) 30°C (1.7x); (f) 20°C (1.8x); (g) 35°C (1.6x); (h) 5% (1.2x); (i) 2% (1.4x); (j) 4% (1.4x); (k) 6% (1.2x); (l) 12 h/12 h (light/dark, 1.9x); (m) 4 h/20 h (light/dark, 1.7x); (n) 24 h light (1.5x); (o) 24 h dark (1.8x); (p) 8 h/16 h (light/dark, 1.6x).

**Figure 5:** (a) Standard gymnemic acid; (b) *in vivo* leaf; (c) OPGRs MS + 2,4-D (1.5 mg/L) with KN (0.5 mg/L); (d) blue light treatment with OPGRs.
